# Radioanatomical Study of the Skull Base and Septum in Chinese: Implications for Using the HBF for Endoscopic Skull Base Reconstruction

This article has been retracted.

**DOI:** 10.1155/2022/9940239

**Published:** 2022-03-29

**Authors:** Dongsheng Gu

**Affiliations:** ^1^Department of Otolaryngology-Head and Neck Surgery, The Affiliated Huaian No. 1 People's Hospital of Nanjing Medical University, Huai'an City, Jiangsu Province, China; ^2^Department of Otolaryngology-Head and Neck Surgery, ENT Hospital of Huaian, Huai'an City, Jiangsu Province, China

## Abstract

**Objective:**

Radioanatomy provides surgeons with different choices to prevent the failure of reconstruction caused by improper flap selection and the occurrence of CSF leakage or other severe complications. To establish a radioanatomical model, this study radioanatomically investigated the use of the Hadad–Bassagasteguy nasoseptal flap (HBF) in skull base reconstruction performed via the transethmoidal, transsphenoidal, and transclival approaches to provide preoperative guidance for the selection of approaches for skull base reconstruction and preparation of the HBF.

**Methods:**

The computed tomography images of 40 Chinese adults were selected for the radioanatomical measurement of data related to the HBF and skull base reconstruction via the transethmoidal, transsphenoidal, and transclival approaches. The results were analyzed using radioanatomy combined with SPSS-based analysis.

**Results:**

In the 40 patients, the area of the HBF exceeded that of skull base defects reconstructed via the transethmoidal approach by 10.21 ± 1.97 cm^2^, and the anterior margin width, posterior margin width, upper margin length, and lower margin lengths of the HBF all exceeded the corresponding values of skull base defects requiring reconstruction by at least 8.4 mm. The area of the HBF exceeded that of reconstructed skull base defects by an average of 10.72 ± 2.04 cm^2^. The area of the HBF exceeded that of skull base defects reconstructed via the transclival approach by 9.01 ± 2.87 cm^2^. The difference between the anterior margin width of the HBF and the middle width of skull base defects reconstructed via the transclival approach did not exceed 6 mm in only one case (5.4 mm).

**Conclusion:**

In Chinese adults, the HBF can cover skull base defects reconstructed via the transethmoidal, transsphenoidal, and transclival approaches, permitting its use in skull base reconstruction performed via all three approaches. Radioanatomy can be used for preoperative guidance to plan surgery via the transethmoidal, transsphenoidal, and transclival approaches.

## 1. Introduction

Endoscopic skull base surgery was initially used to treat pituitary macroadenoma and cerebrospinal rhinorrhea with endoscopic visualization. Currently, it is selectively used to treat lesions located from the frontal sinus to the clivus, including lesions in the anterior, middle, and posterior cranial fossae through the ethmoidal plate, sella turcica/sphenoid bone, and clivus [1, 2]. The development of skull base surgery has been restricted by difficulties with defect reconstruction. Reconstruction of the skull base barrier is conducted to permanently separate the nasal cavity, nasal sinus, and cranial cavity; eliminate postoperative dead space; and protect the physiological functions of the brain as well as important nerves and blood vessels. Therefore, the main challenges of skull base surgery include reconstructing dural defects and preventing cerebrospinal fluid (CSF) leakage [3]. Similar to reconstruction techniques used in open surgery, endoscopic repair must achieve multiple goals: reestablishing the separation between the sterile cranial cavity and nasal cavity colonized by microorganisms, preventing CSF from leaking through the defects, and filling the cavity after tumor resection [3]. The advantages of transcranial endoscopic skull base surgery include low surgical trauma, good tumor exposure, complete resection, and rapid postoperative recovery. The low success of skull base reconstruction is one of the main obstacles preventing the widespread use of transcranial endoscopic skull base surgery [4]. The application of synthetic materials, intranasal and extranasal flaps, and autogenous free tissues in reconstruction after transcranial endoscopic skull base surgery has been reported with good results [5, 6]. Clinicians must increase their mastery of transcranial endoscopic skull base reconstruction because of the high incidence of CSF leakage during and after the surgery. The selection of repair materials and technologies as well as strategies for evaluating these materials has recently become a key area of focus for transcranial endoscopic skull base surgery [7].

In 2006, Hadad et al. [8] firstly designed the Hadad–Bassagasteguy nasoseptal flap (HBF) based on the posterior septal artery, which has been widely used in endoscopic skull base reconstruction. Pinheiro-Neto et al. [9] initially measured the linear data of the anterior skull base, sellar area, and clival area via multiplanar CT image reconstruction and also examined the length, width, and area of the pedicled nasoseptal flap to evaluate whether the tissue flap could completely cover skull base defects created during surgery via different intranasal approaches. A later study by Pinheiro-Neto et al. [10] introduced more parameters in the radioanatomical measurement, improved the selection of measurement markers and methods, expanded the sample size, and increased and improved parameter measurement.

Radioanatomy provides surgeons with different choices to prevent the failure of reconstruction caused by improper flap selection and the occurrence of CSF leakage or other severe complications. To select the proper strategy for skull base reconstruction, preoperative imaging can be used to evaluate the size of tissue flaps and defects. Our study used radioanatomy to explore the clinical significance of the HBF in reconstruction performed after endoscopic skull base surgery. The purpose of this study is to establish a radioanatomical model, carry out the radioanatomical study of HBF and transcribriform, transsphenoidal, and transclival skull base reconstruction, and evaluate the significance of HBF for reconstructing transcribriform, transsphenoidal, and transclival approach skull base defect. It also provides preoperative guidance for the approach size selection for transcribriform, transsphenoidal, and transclival skull base reconstruction and the preparation of HBF.

## 2. Materials and Methods

### 2.1. Clinical Data

Thin-slice axial computed tomography (CT; thickness = 0.3 mm, tube voltage = 110 kV, exposure time = 3.6 s) data of the skull base for 40 adults were used. Inclusion criteria are as follows: in adults (>17 years); including the complete skull base and nasal sinus, which could be used for subsequent MPR using software; exclusion criteria: fractures of the skull base, nasal cavity, or nasal sinus; the presence of tumors and other space-occupying diseases; history of surgery head and face deformities. The included subjects (including 24 women and 16 men) were 21–78 years old (median, 44.5 years). This study was performed in accordance with policies approved by the Ethics Committee of the Affiliated Huaian No. 1 People's Hospital of Nanjing Medical University.

### 2.2. Variables of the Sphenopalatine Foramen (SPF)

After multiplanar reconstruction of CT images, coronal images in which the inferior orbital fissure, pterygopalatine fossa, and SPF were all visible were selected, and the projection points of the SPF in the axial and midsagittal planes were located. Six variables were measured: the distance from the projection point of the SPF to the ipsilateral sphenoethmoidal suture through the infra-anterior sphenoid sinus in the midsagittal position (Figure 1(a)); the distance from the projection point of the SPF to the sphenoethmoidal suture through the base and posterior wall of the ipsilateral sphenoid sinus and then the superior margin of the dorsum sellae in the midsagittal plane (Figure 1(b)); the distance from the projection point of the SPF to the posterior margin of the planum sphenoidale through the base of the sphenoid sinus in the midsagittal plane (Figure 1(b)); the distance from the projection point of the SPF to the vertex of the posterior margin of the dorsum sellae through the base of the sphenoid sinus in the midsagittal plane (Figure 1(b)); the distance from the projection point of the SPF to the vertex of the posterior margin of the clivus through the base of the sphenoid sinus in the midsagittal plane (Figure 1(a)); and the distance from the SPF to the posterior margin of the nasal septum below the anterior wall of the sphenoid sinus in the axial plane (Figure 1(c)). In Figure 1(b), the green line presented the distances from the anterior of planum sphenoidale to tuberculum sellae, the blue line presented the distances from tuberculum sellae to the base of the sphenoid sinus, the red line presented the distances from the top of dorsum sellae to the base of the sphenoid sinus, and the white line presented the distances from SPF to the base of the sphenoid sinus.

### 2.3. HBF Variables

Five HBF variables were measured. The anterior margin width of the HBF was measured as the distance between the anterior nasal spine and rhinion in the midsagittal plane (Figure 2(a)). The posterior margin width of the HBF was measured as the distance from 10 mm below the ethmoidal roof to the nasal floor in the coronal plane (Figure 2(b)). The upper margin length of the HBF was measured as the distance from the rhinion 10 mm below the ethmoidal roof to the anterior wall of the sphenoid sinus in the midsagittal plane (Figure 2(a)). The lower margin length of the HBF was measured as the distance from the lowest end of the nasal septum to the front end of the palatine process of the maxilla in the midsagittal plane (Figure 2(a)). The area of the HBF was measured from the anterior wall of the sphenoid sinus 10 mm below the ethmoidal roof horizontally forward to the posterior wall of the frontal sinus, to the nasal floor forward and downward along the skin mucous junction of the nasal septum, horizontally backward to the posterior margin of the nasal septum, and then to the starting point upward along the anterior wall of the sphenoid sinus (Figure 2(a)). The width of the HBF could be extended to measure the distance between the lateral wall of the nasal cavity under the head end of the inferior turbinate and the nasal septum in the coronal plane (Figure 2(b)).

### 2.4. Variables for Skull Base Reconstruction Performed via the Transethmoidal Approach

Four variables were measured. The anterior margin width was measured as the horizontal distance between the orbital plates of the ethmoid bone at the bilateral anterior ethmoidal foramina in the coronal plane (Figure 3(a)). The posterior margin width was measured as the horizontal distance between the orbital plates of the ethmoid bone at the bilateral sphenoethmoidal sutures in the coronal plane (Figure 3(b)). The defect length was measured as the distance between the frontoethmoidal and sphenoethmoidal sutures in the midsagittal plane (Figure 3(c)). The defect area was measured as the rectangular area of the bilateral orbital plates of the ethmoid bone between the posterior wall of the frontal sinus and the anterior wall of the sphenoid sinus (Figure 3(d)).

### 2.5. Variables for Skull Base Reconstruction Performed via the Transsphenoidal Approach

Seven variables were measured. The anterior margin width was measured as the horizontal distance between the bilateral sphenoethmoidal sutures in the coronal plane (Figure 3(b)). The middle width was measured as the distance between the bilateral optic struts in the coronal plane (Figure 4(a)). The posterior margin width was measured as the distance between the bilateral paraclinoid internal carotid arteries in the coronal plane (Figure 4(b)). The length of the planum sphenoidale was measured as the distance between the sphenoethmoidal suture and the tuberculum sellae in the midsagittal plane (Figure 4(c)). The length of the roof of the sella turcica was measured as the distance between the tuberculum sellae and the upper end of the dorsum sellae in the midsagittal plane (Figure 4(c)). The total length was measured as the distance between the sphenoethmoidal suture and the upper end of the dorsum sellae in the midsagittal plane (Figure 4(c)). The defect area was measured by locating the ethmoidal roof in the midsagittal position and measuring the area forward to the sphenoethmoidal suture and backward to the upper end of the dorsum sellae and bilateral optic strut (Figure 4(d)).

### 2.6. Variables for Skull Base Reconstruction Performed via the Transclival Approach

Five variables were measured. The posterior margin width was measured as the distance between the bilateral paraclinoid internal carotid arteries in the coronal or axial plane (Figure 4(b)). The middle width was measured as the distance between the bilateral internal carotid arteries at the lacerated foramen in the coronal or axial plane (Figure 5(a)). The lower margin width was measured as the distance between the internal margins of the external orifice of the bilateral hypoglossal canals in the coronal or axial plane (Figure 5(b)). The clivus length was measured as the distance between the head end and tail end of the clivus in the midsagittal plane (Figure 5(c)). The clivus area was measured by selecting the long axis section of the clivus in the midsagittal plane in the MPR mode (Figure 5(c)) and reconstructing the images of the clivus (Figure 5(d)). In Figure 5(c), the white dotted line denotes the tangent line of the clivus in the long axis, and the white solid line presents the range from the head end to the tail end of the clivus. Figure 5(d) is the section image of the clivus reconstructed according to the long axis tangent of the clivus, and the area enclosed within the white solid lines corresponds to that enclosed by white solid lines in Figure 5(c).

### 2.7. Radioanatomical Measurement Software

Image Viewer 3.1.14 (Start Technology Co., Ltd., China) was used for radioanatomical measurements, and the measurement results were accurate to 0.1 mm.

Data were input using WPS2019 11.1 (Kingsoft Corp., Zhuhai). Statistical analysis was conducted using SPSS 26.0 (IBM, USA). All values were expressed as the mean ± standard deviation. The normal distribution of data was tested using the Kolmogorov–Smirnov test. Gender differences in data conforming to a normal distribution were analyzed using the independent-samples *t*-test; otherwise, the *χ*^2^ test was used for analysis. Age differences were evaluated using Spearman's correlation analysis. The 95% confidence interval was selected for correlation analyses of gender and age. *P* < 0.05 denoted statistical significance.

## 3. Results

### 3.1. SPF and HBF

The measurement results including SPF and HBF variables are presented in Table 1. Excluding the extensible width of the HBF, all variables exhibited a normal distribution without gender differences as verified using the independent-samples *t*-test (*P* > 0.05). No gender difference was found for the extensible width of the HBF according to the *χ*^2^ test (*P* > 0.05). Spearman's correlation analysis revealed no age differences for any variable (*P* > 0.05).

### 3.2. Skull Base Defects Reconstructed via the Transethmoidal Approach

The average anterior margin width, posterior margin width, defect length, and area of skull base defects reconstructed via the transethmoidal approach are presented in Table 1. Among them, the length of skull base defects reconstructed via the transethmoidal approach through the anterior sphenoid sinus was the sum of the length from the projection point of the SPF to the ipsilateral sphenoethmoidal suture through the infra-anterior sphenoid sinus and the length of skull base defects reconstructed via the transethmoidal approach (the sum of the measured values in Figure 2(a) and Figure 6(c)). The length of skull base defects reconstructed via the transethmoidal approach through the sphenoid sinus was the sum of the length from the projection point of the SPF to the ipsilateral sphenoethmoidal suture through the sphenoid sinus and the length of skull base defects reconstructed via the transethmoidal approach (the sum of the measured values in Figure 2(b) and Figure 6(c)). The mean differences of the data corresponding to HBF are shown in Table 2. All data were normally distributed. The independent-samples *t*-test revealed gender differences in the posterior margin width of skull base defects reconstructed via the transethmoidal approach (*P* = 0.015), the lower margin length of the HBF, and the length of skull base defects reconstructed via the transethmoidal approach (*P* = 0.015), but no gender differences were noted for other variables (*P* > 0.05). Spearman's correlation analysis revealed no age differences for any variable (*P* > 0.05). Using the measured data, we evaluated whether the HBF could completely cover skull base defects reconstructed by the transethmoidal approach. In the 40 patients, the area of the HBF exceeded that of skull base defects reconstructed via the transethmoidal approach by 10.21 ± 1.97 cm^2^, and the anterior margin width, posterior margin width, upper margin length, and lower margin lengths of the HBF all exceeded the corresponding values of skull base defects requiring reconstruction by at least 8.4 mm. Therefore, the HBF could completely cover skull base defects reconstructed via the transethmoidal approach. The total length of the HBF including vascular pedicles was at least 17.6 mm longer than that needed for skull base defect reconstruction via the transethmoidal approach through the anterior sphenoid sinus, but the total length of the HBF including vascular pedicles was 7.02 ± 8.71 mm shorter than that needed for skull base defect reconstruction via the transethmoidal approach through the sphenoid sinus. The HBF could not be used to reconstruct skull base defects via the transethmoidal approach through the sphenoid sinus in any patients. Additionally, the total length of the HBF including vascular pedicles when reconstruction could not be completed in this study and the total length of skull base defects reconstructed via the transethmoidal approach through the sphenoid sinus was analyzed using a scatterplot. The results illustrated that reconstruction requirements were not met in 34/40 (85.0%) cases, and in 33/40 (82.5%) cases, the total length of the HBF including vascular pedicles did not exceed that of skull base defects reconstructed via the transethmoidal approach through the sphenoid sinus (Figure 6).

### 3.3. Skull Base Defects Reconstructed via the Transsphenoidal Approach

The average anterior margin width, middle width, posterior margin width, length of the planum sphenoidale, length of the roof of the sella turcica, total length, and area of skull base defects reconstructed via the transsphenoidal approach are presented in Table 1. The mean differences of the data corresponding to the HBF are shown in Table 2. All data were normally distributed. The independent-samples *t*-test revealed gender differences only for the anterior margin width of skull base defects reconstructed via the transsphenoidal approach (*P* = 0.015). Spearman's correlation analysis revealed age differences for the anterior margin width of the HBF and the anterior margin width of skull base defects reconstructed via the transsphenoidal approach (*P* = 0.040). Using the study data, we evaluated whether the HBF could completely cover skull base defects reconstructed via the transsphenoidal approach. In the 40 patients, the area of the HBF exceeded that of reconstructed skull base defects by an average of 10.72 ± 2.04 cm^2^. The anterior and posterior margin widths of the HBF both exceeded the corresponding values of skull base defects reconstructed via the transsphenoidal approach by at least 10.7 mm. The total length of the HBF including vascular pedicles was 7.8 mm longer than that needed for reconstruction of the planum sphenoidale via the transsphenoidal approach. The anterior margin width of the HBF was at least 5.8 mm wider than that of skull base defects needing reconstruction via the transsphenoidal approach. The total length of the HBF including vascular pedicles was 0.7 mm longer than that needed for reconstruction of the sella turcica via the transsphenoidal approach. The differences between the anterior margin width of the HBF and that of skull base defects requiring reconstruction via the transsphenoidal approach were sorted from low to high using the WPS tool. The difference was 5.8 mm in one case, whereas the value exceeded 6 mm in the remaining cases. The total length of the HBF including vascular pedicles and that needed for reconstruction of the sella turcica via the transsphenoidal approach was analyzed using a scatterplot, as shown in Figure 7. The criterion of a >3 mm difference was achieved for all but three cases. The total length of the HBF including vascular pedicles exceeded that needed for reconstruction of the sella turcica via the transsphenoidal approach in all 40 cases.

### 3.4. Variables of Skull Base Defects Reconstructed via the Transclival Approach

The area of the HBF exceeded that of skull base defects reconstructed via the transclival approach by 9.01 ± 2.87 cm^2^. The difference between the anterior margin width of the HBF and the middle width of skull base defects reconstructed via the transclival approach did not exceed 6 mm in only one case (5.4 mm). The total length of the HBF with vascular pedicles exceeded that required for reconstruction of the skull base defect via the transclival approach by at least 3 mm in all cases (Table 2).

The average upper margin width, middle width, lower margin width, length, and area of skull base defects reconstructed via the transclival approach are presented in Table 1. The mean differences with the corresponding data of the HBF are shown in Table 11. All data were normally distributed. The independent-samples *t*-test revealed no gender differences for any variables (*P* > 0.05). Spearman's correlation analysis revealed that the difference between the posterior margin width of the HBF and the upper margin width of skull base defects reconstructed via the transclival approach was correlated with age (*P* < 0.05), whereas no other correlations with age were identified (*P* > 0.05). Using these data, we evaluated whether the HBF could completely cover skull base defects reconstructed via the transclival approach. In all 40 patients, the area of the HBF exceeded that of skull base defects reconstructed via the transclival approach by 9.01 ± 2.87 cm^2^. The difference between the anterior margin width of the HBF and the middle width of skull base defects reconstructed via the transclival approach did not exceed 6 mm in only one case (5.4 mm). The total length of the HBF including vascular pedicles exceeded that needed for reconstruction of skull base defects via the transclival approach by at least 3 mm in all cases (Table 2).

## 4. Discussion

The success of small skull base defect reconstruction is not related to the technique or tissue used, and thus, tissue flaps with vascular pedicles are not widely used for this purpose [11]. Conversely, large-scale defects require tissue flaps with vascular pedicles [12–14]. Tissue flaps with vascular pedicles provide faster, more reliable, and complete healing, thereby reducing the risk of complications associated with continued communication between the cranial and nasal cavities [15]. At present, the HBF is the most widely used flap clinically. This tissue flap has high toughness and good extendability, and its pedicles can rotate flexibly and cover a large area of skull base defects caused by endoscopic skull base surgery [8]. Currently, the HBF is widely used in endoscopic skull base reconstruction, but little research has assessed its competence for reconstruction. Concerning radioanatomy, the Pinheiro-Neto [16] and Peris-Celda [17] models are two representative radioanatomical models with some common features. It is worth noting that, in theory, the Peris-Celda model provides a more accurate measurement, but it requires curves or polygonal lines, in addition to high requirements for CT image reconstruction in nonstandard planes (both high requirements for CT scanning and postprocessing software), which will affect the accuracy of measurement. The Pinheiro-Neto model is more reliable and permits easier measurements, but its use is limited by difficulty in setting the measuring straight line reasonably in an irregular cavity. Moreover, the possibility of eliminating the dead space using free fat or other grafts is not considered in either model. In this manner, the demand for flap size can be reduced.

At the beginning of this study, we collected a large amount of radioanatomical data to determine the optimal method to measure HBF variables via CT. We measured every variable described in the literature. Considering the repeatability of the measurement results, we used straight lines instead of curves whenever possible. After comprehensive comparison, we chose a quadrilateral area (rectangle and trapezoid) for the measurement. Although the extent to which the HBF is larger than skull base defects in radioanatomy has not been determined, we accepted the standard value of 6 mm [8] and quoted this standard in specific experiments. The model used in our study was extremely likely to underestimate the size of the HBF and overestimate that of skull base defects. First, Peris-Celda et al. [17] found that measurements using straight lines underestimated the increased length of mucosal curves and folds. Second, we adopted a limited model in which some parts of the HBF that can be fully utilized in the clinic might not be included in the measurement. Thus, we chose to design a limited model because overestimating the size of tissue flaps is problematic in clinical application. On the contrary, it is assumed that bones in the whole approach area should be resected for each skull base defect model, whereas only partial resection is needed in the actual surgery. Such a design ensures that mismatches will not occur. Moreover, we designed measurement markers of the model based on the anatomical results and investigated the reconstruction results after changing the route of HBF application by blocking the sphenoid sinus cavity using autogenous free fat.

The vascular pedicle of the HBF is rotatable with a large rotation angle, and its usable surface area covers a wide range. Therefore, it is a commonly used intranasal flap in clinical practice, including uses in the repair and reconstruction of defects in the anterior, middle, and posterior cranial fossae in the midsagittal plane [8, 9]. This flap branches out from its vascular pedicles supplied by the posterior nasal septal artery, which serves as the terminal branch sphenopalatine artery of the maxillary artery. Considering the self-contraction of mucosal flaps, defects are considered to be completely covered when the length and width of the HBF exceeds those of the defect by more than 6 mm and the total length of the tissue flap including pedicles exceeds that of the route of tissue flap implantation for defect reconstruction by 3 mm. If one of these criteria is not met, then the tissue flap is considered to be incompetent for reconstruction [8, 9]. According to the aforementioned criteria and our research results, the length and width of the HBF exceeded those of skull base defects reconstructed via the transethmoidal approach. However, in clinical practice, the extent of opening of the sphenoid sinus during surgery performed via the transethmoidal approach is high [18]. The HBF cannot reach the defect until it passes through the base and posterior wall of the sphenoid sinus and the planum sphenoidale. The total length of the HBF including vascular pedicles cannot meet the lengthened path. The current study results illustrated that the HPF was fully competent for this task in 6/40 patients. Even if the length criterion was adjusted so that the HBF only needed to be longer than the reconstruction length, only seven cases met this standard. Moreover, this result did not differ by age or gender. However, this does not indicate that the HBF is not suitable for the reconstruction of large skull base defects caused by endoscopic skull base surgery performed via the transethmoidal approach. If proper case selection is performed before surgery and the preoperative images of the cases are fully analyzed, then the HBF can be used for skull base defect reconstruction via the transethmoidal approach in some cases [19]. At this time, radioanatomy is particularly important for preoperative surgical planning.

Considering that the anterior margin of the HBF in the horizontal direction is 3 mm wider than that of the defect in practical reconstruction, the anterior margin width of the HBF can completely cover the defect in actual reconstruction [8]. The length difference did not meet the standard requirement of 3 mm in 3/40 cases. Obviously, according to the anatomical findings in the study, this gap is caused by the fact that the HBF can only reach the defect region truly requiring reconstruction through the base and posterior wall of the sphenoid sinus during reconstruction, which can also be solved. Before the surgery, we can evaluate the defect size on CT images according to the range of lesions and surgical approach and examine the size of the required HBF on the images to guide the planning of the surgical approach and design of the HBF.

In the reconstruction of skull base defects via the transclival approach using the HBF, the posterior margin of the HBF covered the upper part of the clivus, and the anterior margin of the HBF covered the end of the clivus defect. On the one hand, the anterior margin of the HBF in the horizontal direction should be 3 mm wider than that of the defect in practical reconstruction. On the other hand, the HBF can also be moved to the tail of the clivus or pushed to the tail of the clivus by blocking the sphenoid sinus, allowing a wider mucosal flap to cover the middle part of the defect. The length and area were sufficient for covering the defects in all 40 cases. Before the surgery, we can evaluate the size of the defect on CT images according to the range of lesions and surgical approach and evaluate the size of the required HBF on the images to guide the planning of the surgical approach and design of the HBF.

According to the aforementioned model design, we conducted this research in three parts. In the first part, gender differences were found for the posterior margin width of skull base defects reconstructed via the transethmoidal approach, the upper length of the HBR, and the length of skull base defects reconstructed via the transethmoidal approach (*P* = 0.015), but no age or gender differences were identified. The results indicate that sphenoid sinus blocking may be necessary, but the effect of sphenoid sinus blocking has been confirmed in clinical practice [20]. The HBF can be used to complete skull base reconstruction via the transethmoidal approach, and radioanatomy can also be used as a guide for preoperative design of the surgical scheme via the transethmoidal approach. In the second part, a gender difference was found for the anterior margin width of skull base defects reconstructed via the transsphenoidal approach (*P* = 0.015), and an age difference was found for the difference between the anterior margin width of the HBF and that of skull base defects reconstructed via the transsphenoidal approach (*P* = 0.040). No other age or gender differences were identified. These findings indicate that sphenoid sinus blocking may be necessary, but the effect of sphenoid sinus blocking has been confirmed in clinical practice [20]. In the third part, an age difference was noted for the difference between the posterior margin width of the HBF and the upper margin width of the defect reconstructed via the transclival approach (*P* = 0.003). No other age or gender differences were observed. Thus, the HBF can be used to complete skull base reconstruction via the transclival approach, and radioanatomy can also be used as a guide for preoperative design of the surgical scheme via the transclival approach. The analysis of gender and age differences was repeated. Therefore, we believe that there are no significant differences related to gender or age overall in the measurement of the HBF and skull base defects reconstructed via the transethmoidal, transsphenoidal, and transclival approaches.

Although the HBF has been widely used in skull base reconstruction in clinical practice and its efficacy is certain, this study also have the deficiencies that the research does not include the content of the HBF in the reconstruction of skull base defects via the transethmoidal, transsphenoidal, and transclival approaches in surgical practice, which also needs to be further developed. In addition, in our study, the HBF area was smaller than the total area of skull base defects reconstructed via the transethmoidal and transsphenoidal approaches in 5/40 cases, smaller than the total area of skull base defects reconstructed via the transsphenoidal and transclival approaches in 16/40 cases, and smaller than the total area of the three defect regions. Therefore, skull base defects caused by transregional or multiapproach surgery will increase significantly when the HBF does not meet the needs of reconstruction.

## 5. Conclusion

This study for the first time performed radioanatomical modeling and systematic radioanatomical analysis of the HBF and skull base defects reconstructed via the transethmoidal, transsphenoidal, and transclival approaches in Chinese adults. The HBF can cover skull base defects reconstructed via the transethmoidal, transsphenoidal, and transclival approaches, and they can be used for skull base reconstruction via all three approaches. Additionally, radioanatomy can be used as a guide for preoperative design of the surgical scheme via the transethmoidal, transsphenoidal, and transclival approaches.

## Figures and Tables

**Figure 1:** Sphenopalatine foramen (SPF) variables. (a) Distances from the SPF to the sphenoethmoidal suture through the anterior sphenoid sinus (solid line) and to the clivus through the base of the sphenoid sinus in the midsagittal plane (dotted line). (b) Distances from the SPF to the sphenoethmoidal suture through the sphenoid sinus (white + blue + green lines), to the posterior margin of the planum sphenoidale through the sphenoid sinus (white + blue lines), and to the upper margin of the dorsum sellae through the sphenoid sinus (white + red lines) in the midsagittal plane. (c) Distance from the SPF to the posterior margin of the nasal septum below the sphenoid sinus in the axial plane.

**Figure 2:** Hadad–Bassagasteguy nasoseptal flap (HBF) variables. (a) The anterior margin width (red line), upper margin length (blue line), lower margin length (white arrow), and area of the HBF (enclosed by solid lines). (b) The posterior margin width (solid line) and extended width of the HBF (dotted line).

**Figure 3:** Measurements in skull base reconstruction performed via the transethmoidal approach. (a) Anterior margin width. (b) Posterior margin width. (c) Length. (d) Area.

**Figure 4:** Variables for skull base reconstruction performed via the transsphenoidal approach. (a) Middle width. (b) Posterior margin width. (c) Planum sphenoidale (solid line), the length of the sella turcica (dotted line), and the total length (solid line + dotted line). (d) Area.

**Figure 5:** Variables for skull base reconstruction performed via the transclival approach. (a) Middle width. (b) Lower margin width. (c) Length (solid line), clivus section (dotted line). (d) Area.

**Figure 6:** The *X*-axis represents the total length of the HBF including vascular pedicles, and the *Y*-axis represents the total length of ASB reconstruction through the sphenoid sinus. The red line (*Y* = *X*) denotes when the total length of the HBF including vascular pedicles was equal to that of ASB reconstruction through the sphenoid sinus. The green line (*Y* = *X* − 3) denotes when the total length of the HBF including vascular pedicles was 3 mm longer than that of ASB reconstruction through the sphenoid sinus.

**Figure 7:** The *X*-axis represents the total length of the HBF including vascular pedicles, and the *Y*-axis represents the total length needed for reconstruction of the sella turcica via the transsphenoidal approach. The red line (*Y* = *X*) denotes when the total length of HBF including vascular pedicles was equal to that needed for reconstruction of the sella turcica via the transsphenoidal approach. The green line (*Y* = *X* − 3) denotes when the total length of the HBF including vascular pedicles exceeded that needed for reconstruction of the sella turcica via the transsphenoidal approach by 3 mm.

**Table 1:** Radioanatomical measurement results (distance, mm; area, cm^2^).

	Overall average	Female average	Male average
Distance from the SPF to the sphenoethmoidal suture through the anterior sphenoid sinus (SPF_SEJ1, mm)	23.02 ± 3.26	23.82 ± 3.27	21.83 ± 2.94
Distance from the SPF to the sphenoethmoidal suture through the sphenoid sinus (SPF_SEJ2, mm)	62.54 ± 7.78	63.75 ± 7.38	60.71 ± 8.24
Distance from the SPF to the posterior margin of the planum sphenoidale through the base of the sphenoid sinus (SPF_P, mm)	47.17 ± 6.78	48.48 ± 6.61	45.20 ± 6.77
Distance from the SPF to the upper margin of the dorsum sellae through the base of the sphenoid sinus (SPF_S, mm)	44.10 ± 5.02	44.73 ± 5.24	43.16 ± 4.68
Distance from the SPF to the clivus through the base of the sphenoid sinus (SPF_C, mm)	29.68 ± 2.88	29.05 ± 2.80	30.62 ± 2.81
Distance from the SPF to the posterior margin of the nasal septum through the anterior sphenoid sinus (SPF_NS, mm)	33.99 ± 3.42	34.36 ± 3.54	33.44 ± 3.26
Anterior margin width of the HBF (HBF_AW, mm)	50.09 ± 3.53	49.57 ± 3.63	50.87 ± 3.35
Posterior margin width of the HBF (HBF_PW, mm)	47.35 ± 3.97	47.38 ± 3.95	47.29 ± 4.14
Upper margin length of the HBF (HBF_UL, mm)	50.62 ± 3.84	49.72 ± 4.15	51.96 ± 2.95
Lower margin length of the HBF (HBF_LL, mm)	46.26 ± 2.62	45.90 ± 2.39	46.78 ± 2.94
Extensible width of the HBF (HBF_W, mm)	12.80 ± 1.89	12.85 ± 1.99	12.73 ± 1.79
Length of the HBF with vascular pedicles (HBF_TL)	84.92 ± 4.79	84.53 ± 4.93	85.50 ± 4.66
HBF area (HBF_S, cm^2^)	19.14 ± 2.20	18.81 ± 2.02	19.65 ± 2.44
Anterior margin width of transethmoidal skull base defects (SKB_E_AW, mm)	25.33 ± 1.84	25.20 ± 1.71	25.53 ± 2.05
Posterior margin width of transethmoidal skull base defects (SKB_E_PW, mm)	26.38 ± 2.84	26.32 ± 2.24	26.46 ± 3.64
Length of transethmoidal skull base reconstruction through the anterior sphenoid sinus (SKB_E_AS, mm)	52.43 ± 5.55	53.44 ± 5.47	50.91 ± 5.50
Length of transethmoidal skull base reconstruction through the sphenoid sinus (SKB_E_PS, mm)	91.94 ± 8.64	93.37 ± 7.53	89.79 ± 9.95
Length of transethmoidal skull base reconstruction (SKB_E_L, mm)	29.40 ± 4.60	29.62 ± 3.87	29.08 ± 5.64
Area of transethmoidal skull base reconstruction (SKB_E_S, cm^2^)	8.93 ± 1.49	8.71 ± 1.36	9.25 ± 1.66
Anterior margin width of transsphenoidal skull base reconstruction (SKB_S_AW, mm)	26.38 ± 2.84	26.32 ± 2.24	26.46 ± 3.64
Middle width of transsphenoidal skull base reconstruction (SKB_S_MW, mm)	28.84 ± 2.37	29.12 ± 2.10	28.41 ± 2.73
Posterior margin width of transsphenoidal skull base reconstruction (SKB_S_PW, mm)	20.13 ± 1.91	19.61 ± 1.63	20.91 ± 2.09
Length of transsphenoidal defects in the planum sphenoidale reconstruction (SKB_S_PL, mm)	15.37 ± 3.36	15.27 ± 3.18	15.51 ± 3.72
Length of transsphenoidal defects in the sellar region reconstruction (SKB_S_SL, mm)	12.42 ± 2.04	11.71 ± 1.67	13.49 ± 2.12
Total length of transsphenoidal skull base reconstruction (SKB_S_TL, mm)	27.79 ± 3.80	26.98 ± 3.42	29.00 ± 4.13
Area of transsphenoidal skull base reconstruction (SKB_S_S, cm^2^)	8.43 ± 1.03	8.24 ± 1.06	8.70 ± 0.96
Anterior margin width of transclival skull base reconstruction (SKB_C_AW, mm)	20.13 ± 1.91	19.61 ± 1.63	20.91 ± 2.08
Middle width of transclival skull base reconstruction (SKB_C_MW, mm)	21.53 ± 2.24	22.01 ± 2.32	20.80 ± 1.96
Posterior margin width of transclival skull base reconstruction (SKB_C_PW, mm)	29.52 ± 3048	28.93 ± 3.00	30.41 ± 4.03
Length of transclival skull base reconstruction (SKB_C_L, mm)	36.78 ± 3.41	36.52 ± 3..08	37.16 ± 3.91
Area of transclival skull base reconstruction (SKB_C_S, cm^2^)	10.13 ± 1.83	10.28 ± 1.96	9.91 ± 1.64

**Table 2:** Differences between HBF variables and those of transethmoidal, transsphenoidal, and transclival skull base reconstructed (distance, mm; area, cm^2^).

	Overall		Female		Male	
	Average	Minimum	Average	Minimum	Average	Minimum
HBF_AW − SKB_E_AW (mm)	24.76 ± 3.84	15.9	24.38 ± 4.11	15.9	25.34 ± 3.45	17.3
HBF_PW − SKB_E_PW (mm)	20.97 ± 4.30	13.7	21.06 ± 3.35	14.9	20.84 ± 5.56	13.7
HBF_UL − SKB_E_L (mm)	21.21 ± 4.70	13.7	20.10 ± 4.40	13.7	22.88 ± 4.77	17.4
HBF_LL − SKB_E_L (mm)	16.85 ± 4.92	8.4	16.29 ± 3.55	10.6	17.70 ± 6.52	8.4
HBF_TL − SKB_E_AS (mm)	32.49 ± 7.46	17.6	31.09 ± 7.92	17.6	34.59 ± 6.38	23.9
HBF_TL − SKB_E_PS (mm)	−7.02 ± 8.71	-20.7	−8.84 ± 7.98	-20.7	−4.29 ± 9.30	-20.3
HBF_S − SKB_E_S (cm^2^)	10.21 ± 1.97	6.3	10.09 ± 1.76	6.3	10.40 ± 2.31	6.2
HBF_AW − SKB_S_AW (mm)	10.91 ± 3.06	5.8	10.40 ± 2.78	5.8	11.69 ± 3.39	6.1
HBF_AW − SKB_S_MW (mm)	18.51 ± 4.74	10.7	18.26 ± 4.35	11.6	18.89 ± 5.39	10.7
HBF_PW − SKB_S_PW (mm)	31.46 ± 4.60	24.2	32.55 ± 4.21	24.5	29.83 ± 4.80	24.2
HBF_UL − SKB_S_TL (mm)	23.14 ± 4.88	14.7	23.19 ± 5.03	14.7	23.06 ± 4.79	14.9
HBF_TL − SKB_PS_TL (mm)	22.38 ± 8.75	7.8	20.78 ± 8.35	8.6	24.79 ± 9.03	7.8
HBF_TL − SKB_ST_TL (mm)	13.03 ± 7.14	0.7	12.82 ± 7.32	2.0	13.34 ± 7.09	0.7
HBF_S − SKB_S_S (cm^2^)	10.72 ± 2.04	6.9	10.56 ± 1.95	6.9	10.95 ± 2.21	7.0
HBF_PW − SKB_(C_AW ) (mm)	31.46 ± 4.60	24.2	32.55 ± 4.21	24.5	29.83 ± 4.80	24.2
HBF_AW − SKB_C_MW (mm)	15.76 ± 3.80	5.4	14.70 ± 3.88	5.4	17.34 ± 3.15	9.8
HBF_AW − SKB_C_PW (mm)	21.21 ± 4.70	13.7	20.10 ± 4.40	13.7	22.88 ± 4.77	17.4
HBF_UL − SKB_C_L (mm)	14.15 ± 4.36	6.1	13.65 ± 4.71	6.1	14.90 ± 3.80	7.5
HBF_TL − SKB_C_TL (mm)	18.46 ± 6.19	6.4	18.95 ± 6.44	6.4	17.72 ± 5.92	9.5
HBF_S − SKB_C_S (cm^2^)	9.01 ± 2.87	3.94	8.53 ± 2.59	3.94	9.74 ± 3.18	5.1

## Data Availability

The labeled dataset used to support the findings of this study are available from the corresponding author upon request.

## References

[1] D, H, Jho, R (1997). Endoscopic endonasal transsphenoidal surgery: experience with 50 patients. *Journal of Neurosurgery*.

[2] Maggiano H., Papay F. A., Dominquez S., Levine H. L., Lavertu P., Hassenbusch S. J. (2010). Rigid endoscopic repair of paranasal sinus cerebrospinal fluid fistulas. *Laryngoscope*.

[3] Jeon C. M., Hong S. D., Seol H. J. (2017). Reconstructive outcome of intraoperative cerebrospinal fluid leak after endoscopic endonasal surgery for tumors involving skull base. *Journal of Clinical Neuroscience: Official Journal of the Neurosurgical Society of Australasia*.

[4] Snyderman C. H., Pant H., Ca Rrau R. L., Prevedello D., Gardner P., Kassam A. B. (2009). What are the limits of endoscopic sinus surgery?: the expanded endonasal approach to the skull base. *Keio Journal of Medicine*.

[5] Kim G. G., Hang A. X., Mitchell C. A., Zanation A. M. (2012). Pedicled extranasal flaps in skull base reconstruction. *Advances in Oto-Rhino-Laryngology*.

[6] Zanation A. M., Thorp B. D., Parmar P., Harvey R. J. (2011). Reconstructive options for endoscopic skull base surgery. *Otolaryngologic Clinics of North America*.

[7] Shahangian A., Soler Z. M., Baker A., Wise S. K., Schlosser R. J. (2017). Successful repair of intraoperative cerebrospinal fluid leaks improves outcomes in endoscopic skull base surgery. *International Forum of Allergy & Rhinology*.

[8] Hadad G., Bassagasteguy L., Carrau R. L. (2006). A novel reconstructive technique after endoscopic expanded endonasal approaches: vascular pedicle nasoseptal flap. *The Laryngoscope*.

[9] Pinheiro-Neto C. D., Prevedello D. M., Carrau R. L. (2007). Improving the design of the pedicled nasoseptal flap for skull base reconstruction: a radioanatomic study. *The Laryngoscope*.

[10] Pinheiro-Neto C. D., Ramos H. F., Peris-Celda M. (2011). Study of the nasoseptal flap for endoscopic anterior cranial base reconstruction. *The Laryngoscope*.

[11] Hegazy H. M., Carrau R. L., Snyderman C. H., Kassam A., Zweig J. (2000). Transnasal endoscopic repair of cerebrospinal fluid rhinorrhea: a meta-analysis. *Laryngoscope*.

[12] (2011). Nasoseptal flap takedown and reuse in revision endoscopic skull base reconstruction. *Laryngoscope*.

[13] Thakur B., Jesurasa A. R., Ross R., Carroll T. A., Mirza S., Sinha S. (2011). Transnasal trans-sphenoidal endoscopic repair of csf leak secondary to invasive pituitary tumours using a nasoseptal flap. *Pituitary*.

[14] Nyquist G. G., Anand V. K., Singh A., Schwartz T. H. (2010). Janus flap: bilateral nasoseptal flaps for anterior skull base reconstruction. *Otolaryngology-Head and Neck Surgery*.

[15] Nobutaka Y., Rhoton A. L. (2005). Vascular anatomy of the anteriorly based pericranial flap. *Operative Neurosurgery*.

[16] Pinheiro-Neto C. D., Snyderman C. H., Fernandez-Miranda J., Gardner P. A. (2011). Endoscopic endonasal surgery for nasal dermoids. *Otolaryngologic Clinics of North America*.

[17] Peris-Celda M., Pinheiro-Neto C. D., Funaki T. (2013). The extended nasoseptal flap for skull base reconstruction of the clival region: an anatomical and radiological study. *Skull Base*.

[18] Fortes F. S. G., Carrau R. L., Snyderman C. H., Kassam A., Gardner P. (2007). Transpterygoid transposition of a temporoparietal fascia flap: a new method for skull base reconstruction after endoscopic expanded endonasal approaches. *Laryngoscope*.

[19] Fortes F. S. G., Carrau R. L., Snyderman C. H. (2007). The posterior pedicle inferior turbinate flap: a new vascularized flap for skull base reconstruction. *The Laryngoscope*.

[20] Wang E. W., Zanation A. M., Gardner P. A. (2019). Icar: endoscopic skull-base surgery. *International Forum of Allergy & Rhinology*.

